The article "Genetic Analysis Reveals Different Mechanisms of IL-5 Involved in the Development of CAD in a Chinese Han Population" was retracted in 2024. Reasons: signs of a paper mill; compromised peer review; unreliable results or conclusions.

# Genetic Analysis Reveals Different Mechanisms of IL-5 Involved in the Development of CAD in a Chinese Han Population

**DOI:** 10.1155/2023/1700857

**Published:** 2023-01-31

**Authors:** Wenjuan Zhang, Junyi He, Meilin Liu, Mingkai Huang, Qianwen Chen, Jiangtao Dong, Hongsong Zhang, Tian Xie, Jing Yuan, Lingfeng Zha

**Affiliations:** ^1^Department of Cardiology, Union Hospital, Tongji Medical College, Huazhong University of Science and Technology, China; ^2^Hubei Key Laboratory of Biological Targeted Therapy, Union Hospital, Tongji Medical College, Huazhong University of Science and Technology, China; ^3^Hubei Provincial Engineering Research Center of Immunological Diagnosis and Therapy for Cardiovascular Diseases, Union Hospital, Tongji Medical College, Huazhong University of Science and Technology, Wuhan 430022, China; ^4^Department of Geriatrics, The Central Hospital of Wuhan, Tongji Medical College, Huazhong University of Science and Technology, Wuhan 430022, China; ^5^Hubei Maternal and Child Health Hospital, Wuhan 430070, China; ^6^Department of Cardiovascular Surgery, Union Hospital, Tongji Medical College, Huazhong University of Science and Technology, Wuhan 430022, China; ^7^Department of Cardiology, Nanjing First Hospital, Nanjing Medical University, Nanjing, China

## Abstract

**Background:**

Coronary artery disease (CAD) is a complex disease and the leading cause of death worldwide. It is caused by genetic and environmental factors or their interactions. Candidate gene association studies are an important genetic strategy for the study of complex diseases, and multiple variants of inflammatory cytokines have been found to be associated with CAD using this method. Interleukin-5 (IL-5) is an important inflammatory immune response factor that plays a role in a various inflammatory disease. Clinical tests and animal experiments indicated that IL-5 is involved in CAD development, but the exact mechanisms are unclear. This study investigated the genetic relationship between the single nucleotide polymorphisms (SNPs) in *IL5* and CAD.

**Materials and Methods:**

Based on the Chinese Han population, we collected 1,824 patients with CAD and 1,920 control subjects and performed a two-stage case-control association analysis for three SNPs in *IL5* (rs2057687, rs78546665, and rs2069812) using the high resolution melt (HRM) technology. Logistic regression analyses were applied to adjust for traditional risk factors for CAD and to perform haplotype and gene interaction analyses. Multiple linear regression analyses were used to study relationships between the selected SNPs and serum lipid levels.

**Results:**

In this study, two-stage case-control association analysis revealed that the allele and genotype frequency distributions of the three *IL5* SNPs were not statistically significant between the case and control groups. In addition, none of the *IL5* haplotypes were associated with CAD. Further stratified analyses were conducted by sex, age, hypertension, and disease status, respectively, and the results revealed that the rs2057687 and rs2069812 of *IL5* were associated with CAD in the male group (*p*_adj_ = 0.025, OR, 0.77 (95% CI, 0.62-0.97); *p*_adj_ = 0.016, OR, 0.82 (95% CI, 0.70-0.97), respectively); the rs2057687 and rs78546665 of *IL5* were associated with late-onset CAD (*p*_adj_ = 0.039, OR, 0.78 (95% CI, 0.62-0.99); *p*_adj_ = 0.036, OR, 1.46 (95% CI, 1.02-1.53), respectively); the rs2069812 of *IL5* was associated with CAD in the hypertension group (*p*_adj_ = 0.036, OR, 0.84 (95% CI, 0.71-0.99)); and none of the SNPs in *IL5* were associated with different CAD states (anatomical CAD and clinical CAD). In addition, the association between SNPs and the serum lipid levels indicated that rs78546665 was positively correlated with triglyceride levels (*p* = 0.012). Finally, SNP-SNP interaction analyses revealed that interactions of rs2057687 and rs2069812 were associated with CAD (*p*_adj_ = 0.046, OR, 0.77 (95% CI, 0.13-4.68)).

The article "Genetic Analysis Reveals Different Mechanisms of IL-5 Involved in the Development of CAD in a Chinese Han Population" was retracted in 2024. Reasons: signs of a paper mill; compromised peer review; unreliable results or conclusions.

**Conclusion:**

This study suggested that the common variants of *IL5* might play a role in CAD by affecting the risk factors for CAD and through SNP-SNP interactions, which provides a new target for specific treatment of CAD patients and a theoretical basis for personalized medicine.

## 1. Introduction

Coronary artery disease (CAD) is a complex cardiovascular disease (CVD) caused by the combined action of genetic and environmental factors. Its pathological basis is coronary atherosclerosis (AS) and/or coronary artery spasm [1, 2]. CAD is one of the leading causes of death worldwide, causing huge economic and medical burdens on society [3]. Currently, the number of patients with CAD in China has reached 11 million [4]. Epidemiological investigations, twin studies, and relative risk studies have shown that there is a significant genetic predisposition to CAD. Compared to people without CAD, relatives of CAD patients have a 2-3.9-fold higher chance of developing CAD [5, 6]. Although genetic studies such as genome wide association studies (GWASs) have found numerous CAD susceptibility genes, these can explain only approximately 28% of the heritability of CAD, which is estimated to be between 40% and 60% [1, 7]. In addition, the specific pathogenic mechanisms underlying a considerable number of CAD susceptibility genes have not been clarified, and researchers still need to determine the genetic basis of CAD using a variety of strategies [8].

The article "Genetic Analysis Reveals Different Mechanisms of IL-5 Involved in the Development of CAD in a Chinese Han Population" was retracted in 2024. Reasons: signs of a paper mill; compromised peer review; unreliable results or conclusions.

Interleukin-5 (IL-5) is a multieffector inflammatory cytokine that plays a role in various diseases by regulating a variety of cells, such as Th2 cells, NK cells, mast cells, B cells, and eosinophils [9]. IL-5 also plays a key role in the development of CVDs. Research has shown that IL-5 can promote the secretion of T15/EO6 IgM antibody and prevent macrophages from absorbing oxidized low-density lipoprotein (ox-LDL) [10], which may explain why selective macrophage overexpression of IL-5 can prevent atherosclerosis from progressing [11]. Sampi et al. tested plasma IL-5 and ox-LDL concentrations in 1,100 middle-aged Finnish individuals in 2008, as well as the human carotid artery intima-media thickness (cIMT) by ultrasound [12]. The results revealed a positive correlation between IL-5 levels and LDL concentrations, while serum IL-5 levels were negatively correlated with cIMT [12]. This is consistent with another study that found a negative correlation between IL-5 and cIMT changes in the common carotid arteries in females [13]. In addition, IL-33 significantly increased IL-5 expression and antioxidant LDL antibodies, whereas administration of IL-5 monoclonal antibody and IL-33 prevented the reduction of atherosclerotic plaque area and the reduction in IL-33-induced ox-LDL antibodies. These findings imply that IL-33 induces IL-5 and LDL antibodies, which may act as a preventive mechanism against atherosclerosis [14].

Single nucleotide polymorphisms (SNPs) of *IL5* have been found to be related to many diseases: for example, rs2069812 on *IL5* was found to be associated with gastric cancer susceptibility in the Polish population [15]. Although existing evidence suggests that IL-5 is involved in atherosclerosis, the genetic relationship between *IL5* and CAD remains unclear. This study investigated the relationship between SNPs of *IL5* and CAD in a Chinese Han population to explore the genetic role of the *IL5* in CAD, so as to gain insight into the role of IL-5 in the development of CAD. To the best of our knowledge, this genetic perspective study is the first to be conducted in a Chinese Han population, providing a theoretical basis for the clinical treatment of CAD.

## 2. Materials and Methods

### 2.1. Study Population

UnionID is a growing database of DNA samples based on the Chinese Han population and is dedicated to explore the molecular genetic mechanisms of various CVDs. At present, the samples in this sample bank are mainly from the Wuhan Union Hospital in the central region of China. All individuals selected for the sample bank signed informed consent forms. The research involved in the sample bank met the requirements of the World Medical Association Declaration of Helsinki and was approved by the local ethics committee of Union Hospital (Wuhan, Hubei) (No. 0157-01). CAD samples and control samples from UnionID were included in our study. The inclusion criteria for CAD samples were [16–18] as follows: (1) coronary angiography of the patient confirmed that at least one main vessel (left main artery, anterior descending branch, circumflex branch, or right coronary artery) was more than 70% narrowed; (2) the patient's history suggested that they had undergone percutaneous coronary intervention (PCI) or coronary artery bypass grafting (CABG); and (3) the patient had a history of myocardial infarction (MI), and the criteria for MI were chest pain for more than half an hour, dynamic ECG changes, and enzymatic changes in levels of creatine kinase isoenzyme (CKMB) and troponin (TNI). Patients with coronary spasm, juvenile hypertension, type 1 diabetes, or congenital heart disease (CHD) were excluded. The inclusion criteria for the control group were as follows: all of whom were over 35 years old without CAD, MI, juvenile hypertension, type 1 diabetes, CHD, rheumatic immune diseases, neoplastic diseases, and stroke. The discovery population comprised 768 CAD samples and 768 control samples. The validation population included 1,056 CAD samples and 1,152 control samples. The combined population consisted of 1,824 CAD samples and 1,920 control samples. Traditional risk factors for CAD include age, sex, body mass index (BMI), hypertension, diabetes mellitus (DM), smoking history, total cholesterol (Tch), triglyceride (TG), high-density lipoprotein cholesterol (HDL-c), and low-density lipoprotein cholesterol (LDL-c), which were all recorded in detail for each participant. The flow chart of the association analysis between IL-5 and CAD is shown in Figure 1.

The article "Genetic Analysis Reveals Different Mechanisms of IL-5 Involved in the Development of CAD in a Chinese Han Population" was retracted in 2024. Reasons: signs of a paper mill; compromised peer review; unreliable results or conclusions.

### 2.2. Tag SNP Selection

LD block maps of the Chinese population covering *IL5* and its upstream and downstream 5 kbp regions were found in the online databases: SNPinfo Web Server (https://snpinfo.niehs.nih.gov/), Ensembl database (http://www.ensembl.org/), and dbSNP (http://www.ncbi.nlm.nih.gov/projects/SNP/). A tag SNP on *IL5* was selected according to the following selection principles: (1) MAF > 0.05 and *r*^2^ > 0.8, (2) preferentially selected SNPs that have been reported to be associated with inflammation in the literature, and (3) preferentially selected SNPs located in the gene promoter and exon regions. Finally, three tag SNPs in *IL5* gene were included in this study: rs2069812, rs78546665, and rs2057687 (Supplementary Table S1).

### 2.3. DNA Extraction and Genotyping

Human peripheral blood genomic DNA was extracted following the instructions of the BloodGen Mini Kit blood gene column small amount extraction Kit (CW 2087). DNA was PCR amplified in a 25 *μ*L reaction system containing 2.5 *μ*L 10x PCR buffer, 0.5 *μ*L dNTPs, 0.5 *μ*L forward and reverse primers (Supplementary Table S2), 1 *μ*L DNA, 1 *μ*L Taq DNA polymerase, 0.5 *μ*L SYTO 9, and 19 *μ*L double-distilled water with TAKARA-TP600 PCR amplifier (Takara, Japan) and genotyped using a Rotor-Gene 6000 High Resolution Melt (HRM) system (Corbett Life Science, Australia). PCR amplification involved preheating at 94°C for 5 minutes, then denaturation at 94°C for 10 seconds, annealing at the optimum temperature for each SNP (59°C for rs2069812, 56°C for rs78546665, and 55°C for rs2057687) for 10 seconds, and extension at 72°C for 15 seconds for 35 cycles. After holding the sample at 72°C for 5 minutes, the endpoint temperature was maintained at 22°C. For HRM genotyping, the peak of allele detection for rs2069812 was 79-83°C, for rs78546665 was 74-78°C, and for rs2057687 was 82-87°C (Supplementary Table S2).

### 2.4. Statistical Analysis

The Hardy-Weinberg equilibrium (HWE) was tested using PLINK software (v.1.07) in the control population. Allelic and genotypic association analyses were conducted using 2 × 2 and 2 × 3 Pearson's chi-squared contingency tables, respectively. Odds ratio (OR) and 95% confidence interval (CI) were calculated using SPSS (v.23.0). Multiple logistic regression was used to adjust for traditional risk factors for CAD, while multiple linear regression was used to assess the effects of SNP genotypes on serum lipid levels (SPSS, v.23.0). Haplotype reconstruction and analysis were performed using Haploview or multiple logistic regression (SPSS, v.23.0). Statistical power analysis and sample size estimation were performed using the Power and Sample Size Calculations program (PS, v.3.0). The statistical power for all SNPs selected in this study was more than 90% with an effect size of 1.3 (HapMap CHB + JPT data), type I error rate alpha was 0.05, and the MAF for rs2057687 is 0.121, for rs78546665 is 0.155, and for rs2069812 is 0.296. The sample size ratio between the control and case groups was 1.

## 3. Results

### 3.1. Population Characteristics

The clinical characteristics of the CAD patients were compared with those of the control group individuals in the discovery, validation, and combined populations (Table 1). The discovery population comprised 768 CAD and 768 control samples. The validation population included 1,056 CAD samples and 1,152 control samples. The combined population consisted of 1,824 CAD samples and 1,920 control samples. The statistical results showed that the trend of each clinical data point in the discovery, validation, and combined groups was consistent. In the combined population, the CAD group's average age, average BMI, proportion of males, and smoking population were significantly higher than those of the control group with *p* value < 1 × 10^−6^. Moreover, the proportion of patients with diabetes and hypertension in the CAD group was significantly higher than that in the control with *p* value < 1 × 10^−6^. Tch, TG, and LDL-c levels in the CAD group were significantly higher than those in the control group with *p* value < 1 × 10^−6^, respectively. The average density of HDL-c in the CAD group was significantly lower than that in the control group with *p* value < 1 × 10^−6^.

The article "Genetic Analysis Reveals Different Mechanisms of IL-5 Involved in the Development of CAD in a Chinese Han Population" was retracted in 2024. Reasons: signs of a paper mill; compromised peer review; unreliable results or conclusions.

### 3.2. Allelic and Genotypic Association Analyses of SNPs in the *IL5* Gene with CAD

None of the three SNPs in *IL5* deviated from the HWE test in the control population (*p* > 0.001). However, in the first phase of the discovery population, the mutant allele frequencies of rs2057687-T, rs78546665-T, and rs2069812-G in the control population were higher than those in the CAD population (in the control population, MAF for rs2057687-T is 0.134, MAF for rs78546665-T is 0.166, and MAF for rs2069812-G is 0.313, while in the CAD population, MAF for rs2057687-T is 0.087, MAF for rs78546665-T is 0.148, and MAF for rs2069812-G is 0.285). rs2057687 was significantly correlated with CAD before correction for traditional risk factors, and the observed *p* value was 7 × 10^−5^. The other two SNPs, rs78546665 and rs2069812, did not correlate with CAD before correction. After correcting for traditional risk factors, rs2057687 was still significantly correlated with CAD (*p*_adj_ = 0.035, OR, 0.68 (95% CI, 0.47-0.97)), but the adjusted *p* values of the other two SNPs were >0.05 (Table 2). In the second-stage validation and combined populations, the three SNPs were not significant after traditional risk factor correction (*p*_adj_ > 0.05) (Table 2).

For genotypic association analysis, in the first phase of the discovery population, rs2057687 was significantly correlated with CAD in both additive (TT/CT/CC) (*p*_obs_ = 3.61 × 10^−4^) and dominant modes (TT+CT/CC) (*p*_obs_ = 7.40 × 10^−5^). After adjusting for traditional risk factors, rs2057687 was significantly correlated with CAD in both additive (TT/CT/CC) (*p*_adj_ = 0.032, OR, 0.67 (95% CI, 0.46-0.97)) and dominant modes (TT+CT/CC) (*p*_adj_ = 0.034, OR, 0.65 (95% CI, 0.44-0.97)). In the second-stage validation and combined population, the three SNPs were not significant in the three analysis modes either before or after risk factor correction, with *p* values > 0.05 (Supplementary Table S3).

The article "Genetic Analysis Reveals Different Mechanisms of IL-5 Involved in the Development of CAD in a Chinese Han Population" was retracted in 2024. Reasons: signs of a paper mill; compromised peer review; unreliable results or conclusions.

### 3.3. Haplotypic and Interaction Analyses between SNPs in the *IL5* Gene and CAD

Haplotype analysis of multiple SNPs is an effective method for association analysis. Haplotype association analysis can provide better insight into the role of a gene in a given disease, with a combination of alleles from all tested SNPs within the gene region. The *IL5* haplotype was constructed using three *IL5* SNPs, and haplotype association analysis was performed in the combined population (Supplementary Figure S1). In our population, eight haplotypes (CGA, CGG, CTA, CTG, TGA, TGG, TTA, and TTG in the order of rs2057687-rs78546665-rs2069812) were detected, in which the CGA haplotype accounted for over 50% of the total haplotypes in the CAD and control populations. The frequency of the TGG haplotype was 9.2% in the control population, higher than 7.6% in the CAD population. Logistic regression analysis indicated that this haplotype was related to CAD before traditional risk factors were corrected, and the observed *p* value was 0.017. The frequency of another haplotype, TGA, was also higher in the control population than in the CAD population, with an observed *p* value of 0.068 as a fair association. However, after the correction for traditional risk factors by multiple logistic regression analysis, none of the eight haplotypes were associated with CAD, and the lowest *p* value was 0.087 (Table 3).

Pairwise interaction analysis of the three SNPs on *IL5* revealed three interactions, one of which was significant. There were eight genotypic combinations in the combined population for which the interaction of rs2057687-TT/rs2069812-AG was correlated with CAD (*p*_adj_ = 0.046, OR, 0.77 (95% CI, 0.13-4.68)) (Table 4). The results for the other two interactions are not presented as no significant results were found.

### 3.4. Delamination Analysis for the Association of SNPs in the *IL5* Gene with CAD Subgroups

Considering that age, sex, and hypertension may have different effects on CAD, the combined population was divided into different subgroups. Patients with CAD were divided into early-onset CAD and late-onset CAD according to the age at onset: early-onset CAD was defined as the age of first onset in males ≤ 55 years and in females ≤ 65 years, while the late-onset CAD was defined as the age of first onset in males > 55 years and in females > 65 years. The study population was divided into hypertensive and nonhypertensive individuals based on whether they had hypertension. Patients with CAD were divided into clinical CAD and anatomical CAD according to the state of the disease: clinical CAD was defined as the occurrence of MI, PCI, CABG, and other surgical treatment, while the anatomical CAD was defined as severe coronary artery stenosis, with coronary angiography indicating that a stenosis degree of at least one main vessel was greater than 70%, regardless of whether MI occurred or whether PCI, CABG, and other surgical treatments were performed. Association analysis was conducted in different subgroups to explore the relationship between SNPs in *IL5* and CAD in these subgroups.

The article "Genetic Analysis Reveals Different Mechanisms of IL-5 Involved in the Development of CAD in a Chinese Han Population" was retracted in 2024. Reasons: signs of a paper mill; compromised peer review; unreliable results or conclusions.

Allelic association analysis showed that rs2057687 and rs2069812 were significantly correlated with CAD in males (*p*_adj_ = 0.025, OR, 0.77 (95% CI, 0.62-0.97); *p*_adj_ = 0.016, OR, 0.82 (95% CI, 0.70-0.97), respectively). The results from the genotypic association analysis showed that rs2057687 was correlated with CAD in males in a dominant mode (TT+CT/CC) (*p*_adj_ = 0.027, OR, 0.76 (95% CI, 0.59-0.97)) and additive mode (TT/CT/CC) (*p*_adj_ = 0.025, OR, 0.77 (95% CI, 0.62-0.97)). rs2069812 was correlated with CAD in males in the additive mode (GG/AG/AA) (*p*_adj_ = 0.018, OR, 0.83 (95% CI, 0.71-0.97)) and recessive mode (GG/AG+AA) (*p*_adj_ = 0.021, OR, 0.67 (95% CI, 0.48-0.94)). rs78546665 was not associated with CAD in males in either allelic or genotypic association analyses. In addition, no SNPs were found to be associated with CAD in females (Table 5).

Allelic association analysis showed that no SNPs were correlated with anatomical CAD or clinical CAD, and the *p* values were not significant either before or after correction (*p* > 0.05) (Table 6). rs2057687 and rs78546665 were associated with late-onset CAD (*p*_adj_ = 0.039, OR, 0.78 (95% CI, 0.62-0.99); *p*_adj_ = 0.036, OR, 1.46 (95% CI, 1.02-1.53), respectively) (Table 7). rs2069812 was correlated with CAD-with-hypertension after correcting for traditional risk factors (*p*_adj_ = 0.036, OR, 0.84 (95% CI, 0.71-0.99)) (Table 7).

### 3.5. Associations between SNPs in the *IL5* Gene and of Serum Lipid Concentrations

Lipids, as independent risk factors for CAD, play a key role in the occurrence and development of CAD. We further explored the relationship between SNPs in *IL5* and serum lipid levels (Tch, TG, HDL-c, and LDL-c). The link between SNPs in *IL5* and serum lipid levels was calculated using a multiple linear regression model in additive, recessive, and dominant modes. However, only in the recessive mode (TT/TG+GG) was rs78546665 positively correlated with triglyceride levels, with a *p* value of 0.012 and a *β* value of 0.282 after correction (Table 8).

## 4. Discussion

This study explored the genetic involvement of IL-5 in CAD by examining the association between SNPs in *IL5* and CAD in a Chinese Han population. We found that the rs2057687 and rs2069812 were associated with CAD in the male group, rs2057687 and rs78546665 were associated with late-onset CAD, rs2069812 was associated with CAD in the hypertension group, and rs78546665 was positively correlated with triglyceride levels. In addition, interactions between rs2057687 and rs2069812 were associated with CAD.

The article "Genetic Analysis Reveals Different Mechanisms of IL-5 Involved in the Development of CAD in a Chinese Han Population" was retracted in 2024. Reasons: signs of a paper mill; compromised peer review; unreliable results or conclusions.

IL-5 is a multifunctional cytokine that stimulates the proliferation, differentiation, and activation of eosinophils and can also induce the differentiation of B and T cells. Previous studies have shown that a variety of inflammatory cells, including macrophages and T lymphocytes, but also mast cells, NK cells, and eosinophils, release IL-5. IL-5 overexpression significantly reduces macrophage and CD4^+^ T lymphocyte infiltration in a mouse acute aortic dissection (AAD) model. Additionally, IL-5 overexpression reduces the levels of IL-1, IL-6, IL-18, and TNF-a in the body [19]. Zhao et al. found that IL-5 overexpression in macrophages reduces AS in LDLR^−/−^ mice [11]. Increased IL-5 levels are found in the plasma of patients with AS, unstable angina, and AMI [20, 21]. IL-5 protein is two times more abundant in the blood of ApoE^−/−^ mice than in ApoE^+/+^ mice [22]. A recent study found no correlation between baseline IL-5 levels and the risk of coronary artery events or stroke after 15.7 ± 6.3 years of follow-up. However, the presence of carotid bifurcation plaques was related to lower IL-5 levels, and a lack of IL-5 promoted plaque growth at the oscillating blood flow site in ApoE^−/−^ mice [23]. Additionally, the antiatherosclerotic effects of valsartan were reduced by anti-IL-5 monoclonal antibody (mAb) therapy, and macrophage infiltration was higher in the anti-IL-5 mAb group than that in the control group [24]. Valsartan treatment reduced the antiatherosclerotic effects without raising blood pressure, indicating that at least in part, valsartan reduced atherosclerosis through enhancing the Th2 immune response [24].

LDL is oxidized during atherogenesis, and new specific epitopes of oxidization arise that can be recognized and responded to by adaptive T cell-dependent (TD) and innate T cell-independent innate type 2 (TI-2) immune cells. The TD immune response produces a large number of TH2 cells, which suppress atherosclerosis by secreting IL-5. In addition, IL-5 stimulates the production and secretion of T15/EO6 IgM via the TI-2 immune response of innate B-1 cells, and T15/EO6 IgM can inhibit the uptake of ox-LDL by macrophages, thus playing a protective role in the development of atherosclerosis [12, 25]. When IL-5 is lacking, the production of T15/EO6 IgM is reduced, leading to accelerated development of atherosclerosis [10]. It was also found that IL-5 levels were negatively correlated with carotid intimal thickness and significantly positively correlated with IgM levels. Plasma IL-5 levels are associated with plasma levels of ox-LDL-binding antibodies and with a reduction in subclinical atherosclerosis in humans [12]. Zhao et al. found that plasma T15/EO6 IgM in mice with specific IL-5 overexpression in macrophages of LDLR^−/−^ mice increased by 58%, and the aortic plaque area and volume decreased by 43% and 2.4 times compared with the control group after 12 weeks of feeding a high-fat diet [11].

The article "Genetic Analysis Reveals Different Mechanisms of IL-5 Involved in the Development of CAD in a Chinese Han Population" was retracted in 2024. Reasons: signs of a paper mill; compromised peer review; unreliable results or conclusions.

Type 2 innate lymphoid cells (ILC2s) are a population of innate cells of lymphoid origin that drive strong type 2 immunity [26]. Mice lacking ILC2 effector cytokines exhibit increased atherosclerosis, and activation of ILC2s is associated with a lower atherosclerotic burden [27]. ILC2s are a potent source of IL-5^28^ and ILC2-derived IL-5 is required to reduce atherosclerosis [27]. As a major source of type 2 cytokines, selective genetic deletion of *ILC2* in LDLR^−/−^ mice accelerates the onset of atherosclerosis, which is avoided by reconstitution with wild type but not IL5^−/−^ ILC2 [28]. ILC2s improve recovery of heart function after MI in mice by promoting cardiac repair. Low doses of IL-2 in patients with ACS activated circulating ILC2s and significantly increased circulating IL-5 levels. IL-2 supplementation in mice increases ILC2 activation and enhances IL-5 secretion, ultimately improving recovery. The protective effect of ILC2s after MI may be due to the production of IL-5 [29].

These findings indicate that IL-5 can inhibit the occurrence of atherosclerosis, and genetic studies have shown that there are CAD susceptibility sites near the *IL5* gene [30]. In our study, the relationship between SNPs of the *IL5* gene and CAD was investigated from a genetic perspective to elucidate its molecular mechanism. We selected three SNPs on *IL5* gene and conducted a two-stage, large sample association analysis in the CAD and control populations of the Han Chinese population and found that these three SNPs were not independently associated with CAD. A previous CAD GWAS meta-analysis from the CARDIoGRAMplusC4D Consortium indicated that rs2057687 and rs2069812 in *IL5* are not associated with CAD of European ancestry [31]. Considering the differences between different disease states, we divided the CAD population into anatomical and clinical CAD populations and found no association between the SNPs and CAD in these two populations. However, when age and sex factors were considered in the analysis, we found that rs2069812 and rs2057687 in *IL5* were associated with CAD in males. It is well known that the incidence of CAD in males is generally higher than that in women, which is most likely related to the presence of more CAD susceptibility sites in males. Recently, sex-specific GWASs displayed a male-specific effect of *IL5* on the mean area of detected carotid plaques [32]. Silveira et al. analyzed plasma IL-5 and its effect on cIMT and found a protective effect of IL-5 in females. In female cervical sections, there is an increasing and substantial negative connection between IL-5 and cIMT [13], and serum IL-5 levels are also associated with other risk factors, such as LDL-c, serum creatinine, fasting plasma glucose, sex, and age [33]. rs2069812 and rs78546665 in *IL5* were associated with late-onset CAD, which is a chronic inflammatory disease in which inflammatory factors play an important role. At different stages of the disease, inflammatory cells selectively secrete cytokines, so the activity of cytokines is a dynamic process. IL-5 may be activated at a later stage and participate in disease development. In addition, in many cases, the mutation does not act directly on the disease, but on the risk factors for the disease, and occurs only when the risk factors are continuously exposed. We further conducted association analysis on two important independent risk factors for CAD and found that rs2069812 was associated with CAD in the hypertensive population, indicating that this SNP was involved in CAD by influencing hypertension. Compared to females with normal blood pressure, females with both hypertensive conditions (gestational hypertension and preeclampsia) exhibited an atherogenic lipid profile at early gestation. However, only those later developing gestational hypertension showed observably elevated serum IL-5 levels [34]. In an association analysis with the lipid profiles, rs78546665 was found to be correlated with total serum cholesterol, indicating that there is a complex and close correlation between the SNPs in *IL5* and blood lipids, which are also involved in the occurrence and development of CAD. Recent studies have found that IL-5 is involved in the lipid metabolism of immune cells and that IL-5 stimulates ABCA1 expression and cholesterol efflux via the miR-211/JAK2/STAT3 signaling pathway in THP-1-derived macrophages [35]. In addition, moderate alcohol consumption decreases serum IL-5 concentrations (∼14%) [36]. In conclusion, the role of a single SNP in *IL5* may lead to CAD by acting on the traditional risk factors for CAD in many ways.

The article "Genetic Analysis Reveals Different Mechanisms of IL-5 Involved in the Development of CAD in a Chinese Han Population" was retracted in 2024. Reasons: signs of a paper mill; compromised peer review; unreliable results or conclusions.

Haplotype analysis can be used to effectively assess the relationship between a group of linked SNPs and diseases or traits. To evaluate the role of *IL5* in CAD, we constructed a haplotype of *IL5* and conducted a haplotype association analysis, but no correlations were found between the *IL5* haplotype and CAD. Furthermore, gene-gene interaction analysis is an effective method for analyzing the effects of interactions between two loci or two genes on traits or diseases. When a trait is controlled by two loci or genes, one locus can mask or increase the effect of the other locus. We further analyzed the influence of the interaction between SNPs of *IL5* on CAD. Through interaction analysis, rs2057687 and rs2069812 were found to be correlated with CAD, while our previous single SNP analysis showed no correlation between a single SNP and CAD, indicating that a single SNP has only a weak effect on CAD. In complex gene regulation networks, association analysis of a single locus may miss the locus truly related to CAD or ignore the influence of gene interactions on disease. Interaction analysis involving multiple loci can provide an understanding of the role of gene regulatory pathways in diseases.

Our study investigated the genetic relationship between *IL5* and CAD in a Chinese Han population. The results showed that the SNPs in *IL5* might play a role in CAD by affecting the traditional risk factors for CAD and through SNP-SNP interactions, providing a new target for the specific treatment of CAD and a theoretical basis for personalized medicine. However, there are still certain limitations to this study. Populations from different areas may be inconsistent due to geographical and living environments, which results in some differences in genetic background and disease susceptibility. However, in this study, our samples, for the most part, were from the Chinese Han population from central China. Studies in North China or other populations should be validated, and more SNPs should be included in further studies. In addition, our study only found the susceptibility SNPs and possible pathogenesis of CAD through statistical methods from the perspective of genetics, which needs further verification by functional experiments.

## Figures and Tables

**Figure 1:** Flow chart of the association analysis between IL-5 and CAD.

**Table 1:** The characteristics of the study population.

Characteristics	Discovery cohort		*p*	Validation-cohort		*p*	Combined cohort		*p*
	CAD (*n* = 768)	Control (*n* = 768)		CAD (*n* = 1056)	Control (*n* = 1152)		CAD (*n* = 1824)	Control (*n* = 1920)	
Age (years)	63.3 ± 11.1	51.6 ± 12.3	<10^−6^	61.7 ± 11.3	57.9 ± 11.8	<10^−6^	62.4 ± 11.2	55.4 ± 12.4	<10^−6^
Male (%)	71.5	59.2	<10^−6^	73.7	50.8	<10^−6^	72.8	54.2	<10^−6^
Smoking (%)	46.5	20.2	<10^−6^	44.6	24.5	<10^−6^	45.4	22.8	<10^−6^
BMI (kg/m^2^)	24.2 ± 1.54	23.7 ± 1.41	<10^−6^	24.4 ± 1.61	23.7 ± 1.41	<10^−6^	24.3 ± 1.58	23.7 ± 1.41	<10^−6^
Hypertension (%)	68.6	14.7	<10^−6^	67.0	44.5	<10^−6^	67.7	32.6	<10^−6^
DM (%)	34.8	4.3	<10^−6^	30.3	13.0	<10^−6^	32.2	9.5	<10^−6^
Tch (mmol/L)	5.09 ± 1.18	4.53 ± 0.90	<10^−6^	5.16 ± 1.16	4.99 ± 1.22	<10^−6^	5.13 ± 1.17	4.81 ± 1.13	<10^−6^
TG (mmol/L)	1.79 ± 1.16	1.45 ± 0.87	<10^−6^	1.82 ± 1.31	1.52 ± 1.01	<10^−6^	1.81 ± 1.25	1.49 ± 0.96	<10^−6^
HDL-c (mmol/L)	1.12 ± 0.29	1.28 ± 0.31	<10^−6^	1.10 ± 0.28	1.30 ± 0.33	<10^−6^	1.11 ± 0.29	1.29 ± 0.32	<10^−6^
LDL-c (mmol/L)	2.98 ± 1.02	2.54 ± 0.72	<10^−6^	3.06 ± 1.08	2.81 ± 0.92	<10^−6^	3.03 ± 1.05	2.70 ± 0.86	<10^−6^

The data are shown as mean ± SD. Categorical data, including gender, smoking status, and other data, were tested using chi-square tests, and measurement data, such as BMI, age, and blood lipid level, were tested using *t*-tests between the cases and controls in each population; CAD: coronary artery disease; DM: diabetes mellitus; BMI: body mass index; Tch: total cholesterol; TG: triglyceride; HDL-c: high-density lipoprotein cholesterol; LDL-c: low-density lipoprotein cholesterol. Age for the case group is the age at diagnosis; age for the control group is the age at enrollment.

The article "Genetic Analysis Reveals Different Mechanisms of IL-5 Involved in the Development of CAD in a Chinese Han Population" was retracted in 2024. Reasons: signs of a paper mill; compromised peer review; unreliable results or conclusions.

**Table 2:** Allelic association analysis between *IL5* and CAD.

Population	SNP allele	*N*		MAF		*p*_hwe_	*p*_obs_	*p*_adj_	OR (95% CI)
		Case	Control	Case	Control				
Discovery	rs2057687^T^	667	729	0.087	0.134	0.793	7 × 10^−5^	0.035	0.68 (0.47-0.97)
	rs78546665^T^	619	692	0.148	0.166	0.259	0.197	0.173	0.81 (0.59-1.10)
	rs2069812^G^	742	745	0.285	0.313	0.224	0.099	0.519	0.93 (0.73-1.07)

Validation	rs2057687^T^	993	1023	0.123	0.119	0.050	0.690	0.661	1.05 (0.84-1.31)
	rs78546665^T^	907	972	0.182	0.165	0.201	0.161	0.157	1.16 (0.95-1.41)
	rs2069812^G^	1039	1017	0.302	0.301	0.020	0.953	0.860	0.99 (0.84-1.15)

Combined	rs2057687^T^	1660	1752	0.108	0.125	0.102	0.030	0.225	0.89 (0.74-1.07)
	rs78546665^T^	1526	1664	0.168	0.166	0.806	0.760	0.674	1.04 (0.88-1.22)
	rs2069812^G^	1781	1762	0.295	0.306	0.011	0.307	0.336	0.94 (0.83-1.07)

SNP: single nucleotide polymorphism; CAD: coronary artery disease; MAF: minor allele frequency; *p*_obs_: observed *p* value; *p*_adj_, *p* value adjusted by the covariates; age, sex, BMI, hypertension, diabetes mellitus, smoking history, Tch, TG, HDL-c, and LDL-c were adjusted; OR: odds ratio after adjustment; *p*_hwe_: *p* value from the Hardy–Weinberg equilibrium tests.

**Table 3:** Haplotype association analysis between *IL5* and CAD.

	Haplotype	*N*		*p*_obs_	*p*_adj_	OR (95% CI)
		Case (%)	Control (%)			
*IL5* gene (rs2057687^T/C^-rs78546665^T/G^-rs2069812^G/A^)	C-G-A	1702 (59.3)	1677 (56.7)	—	—	1
	C-G-G	446 (15.6)	484 (16.4)	0.193	0.087	0.85 (0.71-1.02)
	C-T-A	333 (11.6)	332 (11.2)	0.889	0.681	1.05 (0.85-1.29)
	C-T-G	87 (3.0)	98 (3.3)	0.736	0.980	1.00 (0.69-1.44)
	T-G-A	16 (0.6)	28 (0.9)	0.068	0.191	0.61 (0.29-1.28)
	T-G-G	218 (7.6)	271 (9.2)	0.017	0.184	0.85 (0.67-1.75)
	T-T-A	4 (0.1)	9 (0.3)	0.170	0.361	0.50 (0.12-2.19)
	T-T-G	62 (2.2)	59 (2.0)	0.851	0.872	0.96 (0.61-1.52)

*p*_obs_: observed *p* value; *p*_adj_, *p* value adjusted by the covariates; age, sex, BMI, hypertension, diabetes mellitus, smoking history, Tch, TG, HDL-c, and LDL-c were adjusted; OR: odds ratio after adjustment.

The article "Genetic Analysis Reveals Different Mechanisms of IL-5 Involved in the Development of CAD in a Chinese Han Population" was retracted in 2024. Reasons: signs of a paper mill; compromised peer review; unreliable results or conclusions.

**Table 4:** Interaction analysis between rs2057687 and rs2069812 in *IL5* and CAD under the genotypic model.

Gene/SNP (*n*, case/control)	Types	*N* (%)		*p*_adj_	OR (95% CI)
		Case	Control		
*IL5*-rs2057687^T^/*IL5*-rs2069812^G^ (1640/1628)	TT/GG	16 (1.0)	22 (1.4)	0.125	1.25 (0.53-2.94)
	TT/AG	4 (0.2)	5 (0.3)	0.046	0.77 (0.13-4.68)
	CT/GG	68 (4.1)	61 (3.7)	0.684	1.13 (0.73-1.77)
	CT/AG	226 (13.8)	252 (15.5)	0.177	1.12 (0.86-1.44)
	CT/AA	19 (1.2)	31 (1.9)	0.344	1.49 (0.74-3.01)
	CC/GG	67 (4.1)	93 (5.7)	0.794	1.56 (1.05-2.33)
	CC/AG	416 (25.4)	391 (24.0)	0.499	1.01 (0.81-1.24)
	CC/AA	824 (50.2)	773 (47.5)	—	1

*p*_adj_: *p* value adjusted by the covariates; age, sex, BMI, hypertension, diabetes mellitus, smoking history, Tch, TG, HDL-c, and LDL-c were adjusted; OR: odds ratio after adjustment.

**Table 5:** Allelic and genotypic association analyses of *IL5* with CAD in gender subgroups.

SNP allele	Model	Male			Female		
		*p*_obs_	*p*_adj_	OR (95% CI)	*p*_obs_	*p*_adj_	OR (95% CI)
rs2057687^T^	ALLE	0.007	0.025	0.77 (0.62-0.97)	0.703	0.264	1.20 (0.87-1.65)
	DOM	0.014	0.027	0.76 (0.59-0.97)	0.729	0.279	1.22 (0.85-1.73)
	REC	0.079	0.373	0.68 (0.29-1.60)	0.820	0.630	1.33 (0.42-4.22)
	ADD	0.024	0.025	0.77 (0.62-0.97)	0.932	0.269	1.20 (0.87-1.64)

rs78546665^T^	ALLE	0.619	0.281	1.12 (0.91-1.38)	0.983	0.490	0.91 (0.69-1.20)
	DOM	0.798	0.385	1.11 (0.88-1.40)	0.974	0.663	0.93 (0.67-1.29)
	REC	0.376	0.290	1.46 (0.73-2.91)	0.986	0.376	0.70 (0.31-1.56)
	ADD	0.675	0.278	1.12 (0.91-1.38)	0.999	0.502	0.91 (0.69-1.20)

rs2069812^G^	ALLE	0.040	0.016	0.82 (0.70-0.97)	0.378	0.132	1.18 (0.95-1.45)
	DOM	0.108	0.081	0.83 (0.68-1.02)	0.470	0.137	1.23 (0.94-1.62)
	REC	0.073	0.021	0.67 (0.48-0.94)	0.497	0.454	1.18 (0.76-1.83)
	ADD	0.112	0.018	0.83 (0.71-0.97)	0.695	0.149	1.16 (0.95-1.42)

*p*_obs_: observed *p* value; *p*_adj_: *p* value adjusted by the covariates; OR: odds ratio after adjustment; ADD: additive mode, rs2057687_TT/CT/CC, rs78546665_TT/GT/GG, and rs2069812_GG/AG/AA; DOM: dominant mode, rs2057687_TT+CT/CC, rs78546665_TT+GT/GG, and rs2069812_GG+AG/AA; REC: recessive model, rs2057687_TT/CT+CC, rs78546665_TT/GT+GG, and rs2069812_GG/AG+AA.

The article "Genetic Analysis Reveals Different Mechanisms of IL-5 Involved in the Development of CAD in a Chinese Han Population" was retracted in 2024. Reasons: signs of a paper mill; compromised peer review; unreliable results or conclusions.

**Table 6:** Allelic association analysis of *IL5* with CAD in different disease state subgroups.

SNP allele	CAD-anatomical				CAD-clinical			
	*N* (case/control)	*p*_obs_	*p*_adj_	OR (95% CI)	*N* (case/control)	*p*_obs_	*p*_adj_	OR (95% CI)
rs2057687^T^	1198/1752	0.107	0.361	0.91 (0.74-1.11)	1445/1752	0.026	0.255	0.89 (0.74-1.08)
rs78546665^T^	1096/1664	0.423	0.333	1.09 (0.91-1.30)	1321/1664	0.520	0.467	1.07 (0.90-1.26)
rs2069812^G^	1282/1762	0.237	0.396	0.94 (0.82-1.08)	1544/1762	0.337	0.394	0.94 (0.83-1.08)

CAD-anatomical: CAD subjects with severe coronary stenosis; CAD-clinical: CAD subjects with MI or revascularization; *p*_obs_: observed *p* value; *p*_adj_: *p* value adjusted by the covariates; OR: odds ratio after adjustment.

**Table 7:** Allelic association analysis of *IL5* with CAD in the onset age subgroups and the CAD with hypertension subgroups.

SNP allele	CAD-early-onset		CAD-late-onset		CAD-with-HP		CAD-without-HP	
	*p*_adj_	OR (95% CI)	*p*_adj_	OR (95% CI)	*p*_adj_	OR (95% CI)	*p*_adj_	OR (95% CI)
rs2057687^T^	0.745	1.04 (0.81-1.34)	0.039	0.78 (0.62-0.99)	0.679	0.95 (0.74-1.23)	0.193	0.83 (0.62-1.10)
rs78546665^T^	0.105	0.83 (0.65-1.04)	0.036	1.46 (1.02-1.53)	0.879	1.02 (0.82-1.27)	0.564	1.08 (0.84-1.39)
rs2069812^G^	0.461	0.94 (0.79-1.11)	0.310	0.92 (0.78-1.08)	0.036	0.84 (0.71-0.99)	0.343	1.10 (0.91-1.33)

CAD-with-HP: CAD with hypertension; CAD-without-HP: CAD without hypertension; *p*_adj_: *p* value adjusted by the covariates; OR: odds ratio after adjustment.

**Table 8:** Genotypic association between *IL5* and serum lipid levels.

	Dominant			Recessive			Additive		
	*β*	SE	*p*_adj_	*β*	SE	*p*_adj_	*β*	SE	*p*_adj_
*rs2057687^T^*									
Tch	-0.016	0.048	0.741	-0.140	0.154	0.365	-0.023	0.043	0.584
TG	-0.054	0.045	0.230	-0.215	0.145	0.138	-0.060	0.040	0.137
HDL-c	0.019	0.013	0.142	0.016	0.041	0.685	0.016	0.011	0.154
LDL-c	-0.004	0.036	0.906	-0.060	0.130	0.645	0.001	0.040	0.992
*rs78546665^T^*									
Tch	-0.020	0.044	0.655	0.154	0.120	0.200	0.001	0.038	0.983
TG	0.070	0.036	0.051	0.282	0.113	0.012	0.055	0.041	0.184
HDL-c	-0.011	0.012	0.338	-0.024	0.032	0.456	-0.011	0.010	0.285
LDL-c	0.008	0.032	0.794	0.110	0.102	0.253	-0.004	0.037	0.905
*rs2069812^G^*									
Tch	-0.017	0.038	0.660	0.030	0.064	0.634	-0.004	0.028	0.897
TG	-0.023	0.037	0.535	0.046	0.062	0.455	-0.004	0.028	0.897
HDL-c	-0.002	0.010	0.809	-0.012	0.017	0.468	-0.004	0.008	0.609
LDL-c	-0.002	0.033	0.949	0.013	0.054	0.807	0.002	0.024	0.950

Tch: total cholesterol; TG: triglyceride; HDL-c: high-density lipoprotein cholesterol; LDL-c: low-density lipoprotein cholesterol; ADD: additive mode, rs2057687_TT/CT/CC, rs78546665_TT/GT/GG, and rs2069812_GG/AG/AA; DOM: dominant mode, rs2057687_TT+CT/CC, rs78546665_TT+GT/GG, and rs2069812_GG+AG/AA; REC: recessive model, rs2057687_TT/CT+CC, rs78546665_TT/GT+GG, and rs2069812_GG/AG+AA.

The article "Genetic Analysis Reveals Different Mechanisms of IL-5 Involved in the Development of CAD in a Chinese Han Population" was retracted in 2024. Reasons: signs of a paper mill; compromised peer review; unreliable results or conclusions.

## Data Availability

All data used to support the findings of this study are available from the corresponding author upon request.

## Supplementary Materials

Supplementary Materials Table S1: information for selected tag SNPs of *IL5*. Table S2: primer sequences for PCR and temperature for PCR and genotyping. Table S3: genotypic association analysis between *IL5* and CAD. Figure S1: LD block of *IL5*.
